# An Improved Transformer-Based Neural Machine Translation Strategy: Interacting-Head Attention

**DOI:** 10.1155/2022/2998242

**Published:** 2022-06-21

**Authors:** Dongxing Li, Zuying Luo

**Affiliations:** School of Artificial Intelligence, Beijing Normal University, Beijing 100875, China

## Abstract

Transformer-based models have gained significant advances in neural machine translation (NMT). The main component of the transformer is the multihead attention layer. In theory, more heads enhance the expressive power of the NMT model. But this is not always the case in practice. On the one hand, the computations of each head attention are conducted in the same subspace, without considering the different subspaces of all the tokens. On the other hand, the low-rank bottleneck may occur, when the number of heads surpasses a threshold. To address the low-rank bottleneck, the two mainstream methods make the head size equal to the sequence length and complicate the distribution of self-attention heads. However, these methods are challenged by the variable sequence length in the corpus and the sheer number of parameters to be learned. Therefore, this paper proposes the interacting-head attention mechanism, which induces deeper and wider interactions across the attention heads by low-dimension computations in different subspaces of all the tokens, and chooses the appropriate number of heads to avoid low-rank bottleneck. The proposed model was tested on machine translation tasks of IWSLT2016 DE-EN, WMT17 EN-DE, and WMT17 EN-CS. Compared to the original multihead attention, our model improved the performance by 2.78 BLEU/0.85 WER/2.90 METEOR/2.65 ROUGE_L/0.29 CIDEr/2.97 YiSi and 2.43 BLEU/1.38 WER/3.05 METEOR/2.70 ROUGE_L/0.30 CIDEr/3.59 YiSi on the evaluation set and the test set, respectively, for IWSLT2016 DE-EN, 2.31 BLEU/5.94 WER/1.46 METEOR/1.35 ROUGE_L/0.07 CIDEr/0.33 YiSi and 1.62 BLEU/6.04 WER/1.39 METEOR/0.11 CIDEr/0.87 YiSi on the evaluation set and newstest2014, respectively, for WMT17 EN-DE, and 3.87 BLEU/3.05 WER/9.22 METEOR/3.81 ROUGE_L/0.36 CIDEr/4.14 YiSi and 4.62 BLEU/2.41 WER/9.82 METEOR/4.82 ROUGE_L/0.44 CIDEr/5.25 YiSi on the evaluation set and newstest2014, respectively, for WMT17 EN-CS.

## 1. Introduction

Bahdanau et al. were the first to introduce the attention mechanism to neural machine translation (NMT) along with recurrent neural networks (RNNs): the mechanism weighs the importance of each source token to produce the target token. By contrast, the traditional way predicts each target token in each time step, using the fixed-length context vector [1]. Kalchbrenner et al. [2] and Gehring et al. [3, 4] combined the attention mechanism with models based on the convolutional neural network (CNN) for NMT. Recently, the transformer-based models became fashionable solutions to sequence-to-sequence (seq2seq) problems like NMT [5–7], for they outperform RNN-based models and CNN-based models [1–4, 8, 9]. In every transformer-based model, the encoder-to-decoder structure is adopted to encode the source sequence into a series of hidden representations as the context vector, and the target sequence is then generated based on the context vector [5]. The encoder and decoder are connected through an attention layer.

The transformer-based models, which solely depend on the attention mechanism, outshine the models grounded on RNNs and CNN, thanks to the use of the self-attention network (SAN). In practice, to further improve the expressive power, the transformer-based models employ the multihead self-attention mechanism. Each head projects the input into a lower-dimensional subspace and computes the corresponding attention relationship in that subspace. This projection size for each head is commonly referred to as the head size [10].

However, this multihead attention mechanism has two problems. On the one hand, in theory, more heads make a model more expressive in natural language preprocessing (NLP). However, some scholars demonstrated that more heads do not necessarily lead to better performance. The low-rank bottleneck may arise, once the number of heads surpasses a certain threshold [10]. Namely, more heads generate redundant head information, increase the computational complexity of the model, cause feature redundancy, and reduce performance. Voita et al. [11] and Michel et al. [12] proved that only a small part of the heads is truly important for NMT, especially those in the encoder block. Important heads such as morphology, syntax, and low-frequency words serve multiple functions, while other heads only convey repeated and incomplete information. On the other hand, each head is independent without considering the mutual relationship of all heads. The calculation of each head attention is performed only in the same subspace but not in different subspaces. The multihead self-attention mechanism only concatenates all the results at the end.

To avoid the low-rank bottleneck brought by more heads, Bhojanapalli et al. [10] brought the parameters of the low-dimensional space close to the attention matrix by increasing the key size to the sequence length for a subhead. Shazeer et al. [13] argued that, when the dimension of the subhead reaches the extreme level, the dot product between the query and key does not fit the informational matching function. To address this issue, the talking-head attention emerged. Under this mechanism, the attention can attend to any query and key, regardless of the number and dimensions of the subheads, by learning the linear projection matrices before and after the softmax function. However, both attention mechanisms are also conducted in the same subspace. Besides, the former approach may not improve the machine translation performance, resulting from the varied ranges of sequence lengths. For talking-head attention, more parameters have to be learned, as the attention head distribution becomes more complex.

Therefore, it is necessary to resolve the maximum number of heads for avoiding the low-rank bottleneck and make full use of the interactive information of all heads. To attend to all subqueries and subkeys and prevent the low-rank bottleneck, this paper proposes the interacting-head attention mechanism, based on the following intuitions: (1) when there are relatively few heads, the attention relationship between the head sizes among different subspaces increases with the head size; (2) when there are relatively many heads, the attention relationship between the head sizes among different subspaces decreases with the head size and may be ignored in the most extreme case; (3) the right number of heads must be selected, because it is computationally intensive to calculate the head attention of all tokens in all spaces. The proposed interacting-head attention mechanism enables the head size to talk in the same subspaces and interact with each other in different subspaces. Furthermore, a suitable threshold was defined for the number of heads to control the training time and decoding time, while avoiding low-rank bottleneck and ensuring the head size.

Our model was compared to three baseline multihead attention models on three evaluation datasets. The comparison proves that the interacting-head attention mechanism improves the translation performance and enhances the expressive power. On the dataset IWSLT2016 DE-EN, our model outperformed the original multihead attention model by 2.78 BLEU/0.85 WER/2.90 METEOR/2.65 ROUGE_L/0.29 CIDEr/2.97 YiSi and 2.43 BLEU/1.38 WER/3.05 METEOR/2.70 ROUGE_L/0.30 CIDEr/3.59 YiSi for the evaluation set and the test set, respectively. On the dataset WMT EN-DE, our model outperformed the original model by 2.31 BLEU/5.94 WER/1.46 METEOR/1.35 ROUGE_L/0.07 CIDEr/0.33 YiSi and 1.62 BLEU/6.04 WER/1.39 METEOR/0.11 CIDEr/0.87 YiSi, 1.21 BLEU/6.63 WER/1.42 METEOR/0.51ROUGE_L/0.18 CIDEr/0.52 YiSi, 1.39 BLEU/4.64 WER/0.98 METEOR/5.59 ROUGE_L/0.24 CIDEr/0.42 YiSi, 1.26 BLEU/3.84 WER/1.70 METEOR/0.13 CIDEr/1.30 YiSi for the evaluation set and the newstest2014/2015/2016/2017 test set, respectively. On the dataset WMT EN-CS, our model outperformed the original model by 3.87 BLEU/3.05 WER/9.22 METEOR/3.81 ROUGE_L/0.36 CIDEr/4.14 YiSi and 4.62 BLEU/2.41 WER/9.82 METEOR/4.82 ROUGE_L/0.44 CIDEr/5.25 YiSi, 3.78 BLEU/5.09 WER/9.09 METEOR/4.24 ROUGE_L/0.35 CIDEr/3.97 YiSi, 4.42 BLEU/2.87 WER/3.21 METEOR/4.42 ROUGE_L/0.38 CIDEr/4.83 YiSi, 3.42 BLEU/3.97 WER/2.79 METEOR/3.66 ROUGE_L/0.33 CIDEr/4.00 YiSi for the evaluation set and the newstest2014/2015/2016/2017 test set, respectively.

This research makes the following contributions:

1. Various types of attention mechanisms, which were used in RNNs, CNN, and transformers, were reviewed with mathematical expressions.
2. The authors proposed a method to calculate the maximum number of heads. The method keeps the head size at a large level so that the head attention among the subspaces can be computed well. Moreover, the calculation method solves the low-rank bottleneck and prevents excessively long training and decoding time.
3. For NMT, the interacting-head attention model for the transformer was proposed, under which all attention heads can fully communicate with each other.

## 2. Preliminaries

This section recaps the transformer architecture, which outshines RNNs and CNN in seq2seq tasks, reviews the background of various forms of attention, especially multihead attention used in transformer [5], analyzes the low-rank bottleneck induced by multihead attention in the standard transformer, and introduces the two mainstream solutions to low-rank bottleneck, as well as their problems in NMT.

### 2.1. Transformer

The transformer architecture resolves NMT solely by relying on the attention algorithm [5]. It has been proved that the transformer-based models are superior to the models using RNNs and CNN [1–4, 8, 9]. Like RNNs and CNN, the standard transformer-based model employs the encoder-to-decoder structure for NMT [14]. This structure maps the source sequence to a hidden state matrix as a natural language understanding (NLU) task and views the matrix elements as the context vectors or conditions for producing the target sequence. Encoder and decoder blocks are stacked in the encoder-to-decoder structure.

Each encoder block usually comprises a multihead self-attention layer and a feedforward layer with residual connection [15], followed by a normalization layer [16]. As the core component of the encoder, the multihead self-attention layer captures the hidden representations of all the tokens within the source sequence. This operation mainly depends on the SAN, which learns the mutual attention score of any two tokens in the source sequence. It should be noted that the learned attention scores constitute an asymmetric square matrix, because of the learned parameters. For example, *a*_*ij*_, the attention score from the *i*-th token to the *j*-th token, is not equal to *a*_*ji*_, the attention score from the *j*-th token to the *i*-th token. Specifically, the SAN computes the attention scores by the scaled dot product attention algorithm. Since each token is visible to the others, the encoder can capture the feature of each token in two directions. There are two primary functions of the encoder: (1) learning the hidden representations of the input sequence as a condition for natural language generation (NLG) tasks, for example, NMT; (2) completing downstream NLP tasks, such as sentiment classification or labeling by transfer learning, after being trained independently as a masked language model (MLM) [17] and connected to specific networks.

The decoder blocks have a similar structure as encoder blocks. The only difference lies in an additional sublayer, which computes the attention scores between the representations of the source sequence given by the encoder and the current target token representation given by the multihead SAN of the decoder. This sublayer, known as the encoder-decoder attention layer, is followed by a multihead attention layer. In the decoder, two attention mechanisms, namely, multihead self-attention and encoder-decoder attention, are arranged to capture the hidden state of the target token in each block. Since the token is only visible to its leftward tokens, the self-attention scores form a lower-dimensional triangular matrix. In other words, the multihead self-attention layer aims to focus the current target token only on the leftward tokens and mask the future tokens in the target sequence. In addition, the decoder learns the leftward token representations to generate the token probability distribution in each time step. During training, the probability distribution of the target token is computed based on the ground-truth leftward target tokens or their representations. All the representations are given by the encoder as a context vector for generating the target sequence. During inference, the current token probability distribution is computed based on the previous target token distribution. All the token representations are given by the encoder. The decoder works in a teacher-forcing way during training, while in an auto-regressive way during inference. The difference between the two stages is that the last token feature comes from the last ground-truth token and the last generated token given by the trained model, respectively.

Because the attention mechanism is not order-aware, the transformer-based models add the positional information into the tokens, for example, absolute positional embedding.

### 2.2. Attention

For NMT, the translation performance hinges on the attention mechanism, in addition to the encoder-to-decoder structure. Bahdanau et al. [1] pioneered the use of the attention mechanism for NMT along with RNN. Sutskever et al. [8] and Luong et al. [9] further advanced the implementation of the attention mechanism in NMT. After the introduction of the attention mechanism, a target token no longer depends only on the same context vector. The different roles of the source token in target token generation are reflected. Along with the appearance of the transformer, complicated attention algorithms have been developed for specific NLP tasks, such as single head attention and multihead attention. Apart from linking up the encoder with the decoder, these algorithms learn the relationships in an end-to-end way.

#### 2.2.1. Dot Product Attention

Luong et al. explored the computing methods of an attention score, examined their effectiveness, divided attention mechanisms into global attention and local attention [9] (the former targets all the source tokens, while the latter considers the subset of all the source tokens), and designed three computing methods for the weight scores between two tensors or vectors along with RNNs for NMT. Here, some symbols used in Shazeer et al. [13] are adopted. Three computing methods can be expressed as

(1) $$\begin{array}{c} \text{score}\left(m,x\right)=\begin{array}{c} m^{T}x\text{ dot},\\ m^{T}Wx\text{ general,}\\ \tanh\left(W\left[m,x\right]\right)\text{ concat,} \end{array} \end{array}$$

where *m* ∈ ℝ^*d*^ and *x* ∈ ℝ^*d*^ are the matching and matched column vectors, respectively; *W* ∈ ℝ^*d*×*d*^ is a learned parameter matrix; score(·) is real. The larger the score, the more important *x* is to the generation of *m*. Dot-product attention is widely used for model implementation, by virtue of its fast speed and space efficiency [5]. In line with the notations given by Shazeer et al. [13], the attention between two sequences *X* ∈ ℝ^*n*×*d*^ and *M* ∈ ℝ^*m*×*d*^ is computed through a dot product operation.

(2) $$\begin{array}{c} X=XW_{X},\\ M=MW_{M},\\ \text{Attention}\left(X,M\right)=\text{soft }\max\left(X\cdot M^{T}\right),\\ O=\text{Attention}\left(X,M\right)\cdot M,\\ \hat{O}=O\cdot W_{o}, \end{array}$$

where *n* and *m* are the length of *X* ∈ ℝ^*n*×*d*^ and *M* ∈ ℝ^*m*×*d*^ with the same dimension *d*, respectively. To keep the shape constant between the input and the output, *O* ∈ ℝ^*n*×*d*^ is regarded as the final output or mapped further to a lower or higher dimension with a linear projection matrix *W*_*o*_ ∈ ℝ^*d*×*d*_*o*_^ to get the final output.

#### 2.2.2. Scaled Dot Product Attention

Scaled dot product attention is referred to as single head attention in this research. This attention mechanism projects the input *X* into *d*_*k*_-dimensional queries *Q* and projects the other inputs *M* into *d*_*k*_-dimensional keys *K* and *d*_*v*_-dimensional values *V*. The increase of *d*_*k*_ pushes up the dot products, which in turn make the softmax function converge into regions where it has extremely small gradients [5]. Therefore, the attention score is scaled with $1/\sqrt{d_{k}}$.

Firstly, it is necessary to explain the calculation of attention scores by a single head attention between two tensors *X* ∈ *ℝ*^*n*×*d*_*X*_^ and *M* ∈ *ℝ*^*m*×*d*_*M*_^, where the next projection operation is needed to deal with the dimensional difference. The matrices of queries *Q* ∈ *ℝ*^*n*×*d*_*k*_^, keys *K* ∈ *ℝ*^*m*×*d*_*k*_^, and values *V* ∈ *ℝ*^*m*×*d*_*v*_^ can be, respectively, obtained with the linear projection matrices *W*_*q*_ ∈ *ℝ*^*d*_*X*_×*d*_*k*_^, *W*_*k*_ ∈ *ℝ*^*d*_*M*_×*d*_*k*_^, and *W*_*v*_ ∈ *ℝ*^*d*_*M*_×*d*_*v*_^ on *X*, M, and M. The global computing can be defined as

(3) $$\begin{array}{c} Q=X•W_{q},\\ K=M•W_{k},\\ V=M•W_{v},\\ \text{Attention}\left(X,M\right)=\text{soft }\max\left(\frac{QK^{T}}{\sqrt{d_{k}}}\right),\\ O=\text{Attention}\left(X,M\right)•V,\\ \hat{O}=O•W_{o}, \end{array}$$

where **O** ∈ *ℝ*^**n**×**d**_**v**_^ is the output. The $\hat{O}$ value is obtained following the last linear projection. If the self-attention scores are computed within a sequence, the linear projection matrices **W**_**q**_, **W**_**k**_, **W**_**v**_, and**W**_**o**_ must function on the same tensor; namely, **X** ≡ **M**. If **X** is different from **M**, the encoder-to-decoder attention scores should be calculated by the formula (3). Scaled dot production self-attention is applied in the SAN of the encoder and the decoder, as well as the encoder-decoder attention layer. In fact, Vaswani et al. [5] used a transformer to capture the token dependencies, relying on multihead scaled dot production attention.

#### 2.2.3. Multihead Attention

In the standard transformer, it is beneficial to split the representations into multiple heads and concatenate the subresults of heads in the end. This is because more heads elevate the expressive power and improve model performance. Both tensors are employed on **X** ∈ *ℝ*^**n**×**d**_**X**_^ and **M** ∈ *ℝ*^**m**×**d**_**M**_^, where **X** represents the matching tensor and **M** represents the matched objective. The dimensions of queries, keys, and values are then split into *h* parts, which is equal to the number of heads. Therefore, the two tensors can be projected into three low-dimensional matrices (subqueries, subkeys, and subvalues) with the corresponding low-dimensional parameter matrices **W**_**q**_^**i**^ ∈ *ℝ*^**d**_**X**_×**d**_**k**^**i**^_^, **W**_**k**_^**i**^ ∈ ℝ^**d**_**M**_×**d**_**k**^**i**^_^, and**W**_**v**_^**i**^ ∈ *ℝ*^**d**_**M**_×**d**_**v**^**i**^_^ for the **i** − **th** head. Under most circumstances, **d**_**k**^**i**^_ is equal to **d**_**v**^**i**^_, and both are set to **d**/**h**, with **d** being the model dimension [5].

In the end, all the suboutputs **O**^**i**^ ∈ *ℝ*^**n**×**d**_**v**^**i**^_^ of subhead **h**_**i**_ are concatenated as the final result **O** ∈ *ℝ*^**n**×**d**_**v**_^. The final result can be further mapped into a lower or higher dimension with a linear projection matrix **W**_**o**_ ∈ *ℝ*^**d**_**v**_×**d**_**o**_^.

(4) $$\begin{array}{c} Q^{i}=X•W_{q}^{i},\\ K^{i}=M•W_{k}^{i},V^{i}=M•W_{v}^{i},\\ {\text{Attention}}^{i}\left(X,M\right)=\text{soft}\max\left(\frac{Q^{i}{\left(K^{i}\right)}^{T}}{\sqrt{d_{k^{i}}}}\right),\\ O^{i}={\text{Attention}}^{i}\left(X,M\right)•V^{i},\\ O=\text{Concat}{\left[O^{i}\right]|}_{i=1}^{h},\\ \hat{O}=O•W_{o}. \end{array}$$

In the standard transformer, the multihead attention mechanism is utilized in three sublayers: encoder SAN, decoder SAN, and encoder-decoder attention. During model implementation, all three sublayers adopt multihead dot product attention.

### 2.3. Low-Rank Bottleneck of Multihead Attention and Current Solutions

#### 2.3.1. Low-Rank Bottleneck

More heads theoretically enhance the expressive power, and fewer heads mean weaker expressive ability. Nevertheless, Bhojanapalli et al. [10] found when the number of the heads is greater than **d**/**n** (**d** and **n** are the model dimension and the sequence length, respectively), a low-rank bottleneck appears, making the model unable to represent an arbitrary context vector. To remove the bottleneck, the dimension d of the model can be increased while increasing the head number. This approach is obviously expensive because more memory resources are required for the intense computations for model training.

#### 2.3.2. Increasing Key Size and Head Size

The **Q**, **K,**and**V** are always set in the same dimensions (**d**). After determining the model dimension *d* and the number of heads **h**, a subhead projects **Q**, **K,**and**V** into some subspaces of **Q**^**i**^ ∈ *ℝ*^**n**×**d**_**k**^**i**^_^, **K**^**i**^ ∈ *ℝ*^**n**×**d**_**k**^**i**^_^,and**V**^**i**^ ∈ ℝ^**n**×**d**_**v**^**i**^_^, using a series of projection matrices **W**^**i**^ ∈ ℝ^**d** × **d**/**h**^, where *n* represents the length of the sequence, and **d**_**k**^**i**^_=**d**_**v**^**i**^_=**d**/**h** is the subdimension. Then, the **i** − **th** head attention computes with $\mathrm{Atte}n^{i}=\mathrm{soft}\;\max\left(Q^{i}{\left(K^{i}\right)}^{T}/\sqrt{d_{k^{i}}}\right)$ to produce a self-attention square matrix **Atten**^**i**^ ∈ *ℝ*^**n**×**n**^. Finally, the suboutputs **O**^**i**^ ∈ *ℝ*^**n**×**d**_**v**^**i**^_^ of the dot product between **Atten**^**i**^ and **V**^**i**^ are concatenated.

Nonetheless, projecting into a low-dimension subspace is equivalent to mapping a **n**^2^-dimension attention score matrix with 2**n** · **d**/**h** variables. With the increase of **h**, 2**n**•**d**/**h** ≪ **n**^2^ results in a low-rank bottleneck. It is not ideal to reduce **h** or increase **d**. Either of them reduces the expressive power or adds to the computing load. Bhojanapalli et al. [10] presented a solution that breaks the constraint of **d**_**k**^**i**^_=**d**_**v**^**i**^_=**d**/**h**: 2**nd**_**k**^**i**^_⟶**n**^2^ is realized by increasing the key size **d**_**k**^**i**^_. This approach, without changing the shape of the attention head or the computing process, satisfies the following relationships:

(5) $$\begin{array}{c} d_{k^{i}}=n,\\ d_{k^{i}}\neq d_{v^{i}},\\ d_{v^{i}}=\frac{d}{h}. \end{array}$$

#### 2.3.3. Talking-Head Attention

According to Vaswani et al., adequately increasing the size of heads could improve the expressive power. But this is not supported by any empirical evidence [5]. Specially, the translation is rather poor, when the token embedding is reduced to just one scalar. Under this circumstance, the dot product of the queries (one scalar) and keys (one scalar) cannot represent their subspace features. Shazeer et al. put forward a variant of multihead attention called talking-head attention, which adds two linear transformation matrices before and after the softmax function to compute the attention weights of the **i** − **th** head [13]. The addition enables each attention head to talk with each other.

(6) $$\begin{array}{c} Q^{i}=X\cdot W_{q}^{i},\\ K^{i}=M\cdot W_{k}^{i},\\ V^{i}=M\cdot W_{v}^{i},\\ J^{i}=\frac{Q^{i}\cdot {\left(K^{i}\right)}^{T}}{\sqrt{d_{k^{i}}}},\;i\in \left[1,h\right]. \end{array}$$

In talking-head attention, the attention score of the **i** − **th** head **J**^**i**^ ∈ *ℝ*^**n**×**m**^ is calculated the same as multi-head attention. Before normalization with the softmax function, the first talking between all heads is established with the projection matrix **W**_**t**1_ ∈ *ℝ*^**h**×**h**^.

(7) $$\begin{array}{c} J={\left[J^{i}\right]|}_{i=1}^{h},\\ \hat{J}=W_{t1}\cdot J. \end{array}$$

Then, normalization is performed to get the attention weight, using the softmax function. After that, the second talking is established with another projection matrix **W**_**t**2_ ∈ *ℝ*^**h**×**h**^.

(8) $$\begin{array}{c} A^{i}\left(X,M\right)=\text{soft }\max\left({\hat{J}}^{i}\right),\\ A={\left[A^{i}\right]|}_{i=1}^{h},\\ {\hat{J}}^{-1}=W_{t2}\cdot A. \end{array}$$

At last, the final output representations for **X** are computed by the same method as multihead attention.

(9) $$\begin{array}{c} O^{i}={\left({\hat{J}}^{-1}\right)}^{i}\cdot V^{i},\\ O={\left[O^{i}\right]|}_{i=1}^{h},\\ \hat{O}=O\cdot W_{o}. \end{array}$$

#### 2.3.4. Defects of the Two Solutions

The first solution aims to make 2**n** · **dk**⟶**n**^2^ or **dk**⟶**n**. The designers of the solution set the head size of a head attention unit to the input sequence length and defined it as independent of the number of heads. For NMT, however, the sequence length varies greatly. The second solution employs linear transformation to change the distribution of different subattention matrices, which significantly increases the number of trainable parameters. In addition, the increase of **h** reduces the value of **d**_**k**_ and weakens the features generated by the subspace. As a result, the second solution cannot improve the final translation performance. Overall, the low-rank bottleneck cannot be effectively solved, unless more complex high-dimensional spatial transformations are called for help.

## 3. Interacting-Head Attention

### 3.1. Theoretical Hypothesis

In the original multihead attention, a subhead computes the dot product among the subembeddings (head size) of the tokens in the same subspace. The head size in different subspaces is expected to have a strong correlation. The correlation should be strong when the head size is large or the number of heads is small and weak when the head size is small or the number of heads is large. The subembedding of different subspaces can be ignored because the subembedding of the same subspace is very small. Obviously, when the head size limitation reaches 1 and the number of heads equals model dimension, the dot product of subembedding in the same subspace is equal to the product of two scalars. This certainly cannot express the feature information of the same subspace. To calculate the correlation of the head size in different subspaces, this paper proposes a novel attention mechanism called interacting-head attention. It is assumed that the head size is no greater than the sequence length, aiming to prevent the low-rank bottleneck. The effectiveness of our model was verified experimentally based on this hypothesis.

To clarify the composition, the associations between two adjacent tokens with different head sizes in different subspaces are displayed in Figure 1, where the red line indicates the association of the head size in the same subspace, and the blue, black, green, and brown lines specify the association of the head size in subspaces 1, 2,…, (*h* − 1) and *h*, respectively. In fact, there is an association between any two head sizes of the tokens in different subspaces.

### 3.2. Graphical Representation

As shown in Figure 2, the traditional multihead attention adopts the method of dividing before combining. Each subhead represents the matching between subembeddings in the same subspace. However, not all subheads are associated with each other. If the number of heads grows, the omission of the dependency among some heads will result in low performance. What is worse, only the partial attention among the corresponding queries and keys is considered, although the traditional mechanism covers the main matching information. In contrast, our mechanism considers the dependencies of all the attention among the queries and keys. In addition, it is assumed that the different dimensions of the head size of a token indicate morphology, syntax, and semantic information, respectively. The morphology must also have a close association with the morphology (more important attention score) of other tokens. Needless to say, it is also related to the syntax and semantic information of other tokens.

Our mechanism has the following advantages:

1. Compared with talking-head attention, our mechanism does not need to learn extra parameters, and only adds some inner product computations.
2. Our mechanism learns subordinate information by interacting-head attention, in addition to the attention computation of all the tokens with talking-head attention in the same subspace. In this way, all parts can fully communicate with each other.

### 3.3. Sufficient Interactions between Heads

To ensure that any attention head attends to all subqueries and subkeys, this paper further examines the relationship between any subquery from the matching tensor **X** ∈ *ℝ*^**n**×**d**_**X**_^ and all the subkeys from the matched tensor **M** ∈ *ℝ*^**m**×**d**_**M**_^, where **X** and **M** are the feature matrices of the source and target sequences, **n** and **m** are their lengths, and **d**_**X**_ and **d**_**M**_ are their dimensions, respectively. It is assumed that the number of heads is set to **h**. Like the original multihead attention, for the *i*th subspace, both tensors are mapped to other tensors **Q**^*i*^, **K**^*i*^, **V**^*i*^ with the lower dimension using three linear transformation matrices **W**_**q**_^**i**^, **W**_**k**_^**i**^, and **W**_**v**_^**i**^. Actually, the dimensions of **W**_**q**_^**i**^ ∈ *ℝ*^**d**_**X**_×**d**_**k**^**i**^_^ and **W**_**k**_^**i**^ ∈ *ℝ*^**d**_**M**_×**d**_**k**^**i**^_^ must be equal for resolving the dot product. Otherwise, **W**_**v**_^**i**^ ∈ *ℝ*^**d**_**M**_×**d**_**v**^**i**^_^ is the linear transformation matrix for **M** with **d**_**k**^**i**^_=**d**_**v**^**i**^_=**d**/**h**. This process can be expressed as

(10) $$\begin{array}{c} Q^{i}=X\cdot W_{q}^{i},\\ K^{i}=M\cdot W_{k}^{i},\\ V^{i}=M\cdot W_{v}^{i},\;i\in \left[1,h\right]\\ Q^{i}\in {\mathbb{R}}^{n\times d_{k^{i}}},\;K^{i}\in {\mathbb{R}}^{m\times d_{k^{i}}},\;V^{i}\in {\mathbb{R}}^{m\times d_{v^{i}}}. \end{array}$$

For **Q**^**i**^, the attention scores between it and all the subkeys are computed and then normalized by the softmax function.

(11) $$\begin{array}{c} {\text{Attention}}_{ij}\left(X,M\right)={\text{soft }\max\left(\frac{Q^{i}{\left(K^{j}\right)}^{T}}{\sqrt{d_{k^{i}}}}\right)|}_{\text{j}=1}^{h},\\ O^{ij}={{\text{Attention}}_{ij}\left(X,M\right)\cdot V^{j}|}_{j=1}^{h}, \end{array}$$

where **O**^**ij**^ ∈ *ℝ*^**n**×**d**_**v**^**i**^_^ is the attention output between the special subquery *Q*^*i*^ and the dynamic subkey *K*^*j*^. Assuredly, the calculation of the interacting-head attention on one sequence only needs to replace **M** with **X**. Next, the final output **O** can be obtained through similar concatenations of sub-sub-output and sub-output, respectively:

(12) $$\begin{array}{c} O^{i}={\text{concat}\left[O^{ij}\right]|}_{j=1}^{h},\\ \text{axis}=-1,\\ O=\text{concat}\left[O^{i}\right]\cdot W_{o}. \end{array}$$

A minimal python implementation is shown in Algorithm 1. In practice, the deep learning framework keras is used for all our experiments.

### 3.4. Choosing the Suitable Number of Heads

In Section 2.2.3, the dimensions of the **Q**^**i**^, **K**^**i**^, and**V**^**i**^ matrices of the *i*th head are subject to **d**_**q**^**i**^_=**d**_**k**^**i**^_=**d**_**v**^**i**^_=**d**/**h**, which can be written as h=**d**/**d**_**k**^**i**^_. According to the definition of head size in [10], it can be expressed as *h*=**d**/**d**_**k**^**i**^_=**d**/head_size. As mentioned before, increasing model dimensionality and the number of heads can enhance the expressive ability. But a heavy computing load and a large memory demand will ensue, which lead to a low-rank bottleneck. Our model initially adopts a fixed dimensionality *d*. Inspired by [10], to prevent the low-rank bottleneck, the sequence length is regarded as the minimum head size. Therefore, the mean sequence length of the training set should be computed to obtain the maximum number of heads. In our model, the maximum possible number of heads is computed by

(13) $$\begin{array}{c} h_{\max}=\frac{d}{\text{head}\_\text{size}}=\frac{d}{n}, \end{array}$$

where *d* is the model dimensionality and *n* is the mean sequence length of the training set.

## 4. Experiments

This section tests our model on three datasets, namely, IWSLT16 DE-EN, WMT17 EN-DE, and WMT17 EN-CS. All of them are widely used as NMT benchmarks. Before the experiments, the three datasets were preprocessed, and the hyperparameters were configured. Three classic and efficient models were selected as baselines to demonstrate the superiority of our model in translation quality. The experimental results were analyzed to verify our hypothesis and reveal the merits and defects of our model.

### 4.1. Datasets

For the IWSLT16 DE-EN corpus, the experimental data were extracted from the evaluation campaign of the International Conference on Spoken Language Translation (IWSLT 2021) [18]. The extracted data consist of 181 k/12 k sentence pairs as training/evaluation sets. The concatenation of tst2010/2011/2012/2013/2014 was taken as the test set, including around 12 k sentence pairs.

For the WMT17 machine translation task, EN-DE and EN-CS MT tasks were chosen as our problems because of the limited memory resources [19, 20]. For WMT17 EN-DE and EN-CS corpora, the training set consists of 5.85 million and 1 million sentence pairs, respectively. For the two corpora, newstest2013 of 3 k sequence pairs was treated as our evaluation set and newstest2014/2015/2016/2017 as the test set.

Both datasets were preprocessed through data normalization and subword segmentation, using Moses, a de-facto standard toolkit for statistical machine translation (SMT) [21]. Firstly, the sentence pairs of all datasets were tokenized, and those longer than 80/80/100 on the training sets of IWSLT16 DE-EN, WMT17 EN-CS, and WMT17 EN-DE, respectively, were discarded. After that, a truecase model was trained on the cleaned train set and applied to each subset. Secondly, all sequence pairs were encrypted by bytes pair encoding (BPE) [22], using a sentence piece tool (https://github.com/google/sentencepiece) [23]. This step mitigates the influence of unknown (UNK), padding (PAD), and rare tokens. In IWSLT16 DE-EN and WMT17 EN-DE translation tasks, the source and target languages (EN and DE) have similar alphabets. Therefore, a shared vocabulary with 40,000/80000 tokens was learned on IWSLT16 and WMT17, respectively. In the WMT17 EN-CS translation task, a vocabulary was learned for English (EN) and Czech (CS) separately, because the two languages are distant from each other.

As can be seen from Table 1 and Figure 3, the sequence lengths of the languages in different datasets obeyed similar distributions and remained consistent with the mean sequence lengths. The length of sequence ranged from 3 to 120, from 1 to 332, and from 1 to 316 for IWSLT16 DE-EN, WMT17 EN-DE, and WMT17 EN-CS, respectively. The mean sequence lengths of the three datasets were set as 20, 25, and 26, respectively.

### 4.2. Parameter Settings

The settings of our experimental parameters refer to those in [5] which first proposed the transformer architecture for NMT. Our experiments were arranged based on an appropriate setup on the optimizer, learning rate, and hyperparameters. The optimizer was designed by Adam with *β*_1_=0.9, *β*_2_=0.997, and *ε*=10^−9^ as our optimizer [24]. The learning rate was configured by the warm-up strategy [5] with warm up − steps=8000. During training, the label smoothing rate [25] was set to 0.1, and the dropout was fixed at 0.1. Moreover, because of the limitation of GPU memory, the dimension of the hidden state for linear transformation was set to 1024, and the model dimension was set to 512. To avoid the low-rank bottleneck, the maximum number of heads was obtained by formula (13).  Table 2 lists the possible values of the number of heads.

All the experiments were conducted with TensorFlow 1.4.1 and keras 2.1.3 with reference project (https://github.com/Lsdefine/attention-is-all-you-need-keras). The attained model cpt files can also be converted into PyTorch bin files with transformers [26]. All the experiments were completed by two NVIDIA Tesla V100 GPUs of 32 GB memory.

During the inference, a beam search algorithm was used with beam size 4 and batch size 8 to decode all test sets. The length penalty was set to 1 and 0.6 for IWSLT16 and WMT17 test sets, respectively.

### 4.3. Evaluation Metrics

The machine translation quality was evaluated objectively by multiple metrics, including bilingual evaluation understudy (BLEU) [27], word error rate (WER) [28], metric for evaluation of translation with explicit ordering (METEOR) [29], recall-oriented understudy of gisting evaluation (ROUGE) [30], consensus-based image description evaluation (CIDEr) [31]and YiSi [32].

1. BLEU [27]. BLEU, one of the most manifold evaluation methods for machine translation, uses N-gram token matching to evaluate the similarity between the reference and the candidate. The quality is positively correlated with the proximity between the translations and the references.
2. WER [28]. Similar to translation edit rate (TER) [33], WER computes the word error rate between the reference and hypothetical translation. The word errors include the number of substitutions, insertions, and deletions from the translation to the reference. The rate is the ratio of word errors to the length of the reference.
3. METEOR [29]. Based on explicit word-to-word matches, METEOR includes identical words in the surface forms, morphological variants in stemmed forms, and synonyms in meanings between the reference and the candidate.
4. ROUGE [30]. ROUGE was introduced by Chin-Yew Lin for text summarization. It contains four different measures: ROUGE-N, ROUGE-L, ROUGE-W, and ROUGE-S. Here, ROUGE-L is selected as the metric to evaluate machine translation. Note that *L* is the abbreviation of the longest common subsequence (LCS) between the reference and the candidate.
5. CIDEr [31]. CIDEr is originally used to evaluate the generated image descriptions. It measures the similarity of a generated sequence against a set of ground truth sentences written by humans. This similarity reflects how well the generated descriptions capture the information of grammaticality, saliency, importance, and accuracy.
6. YiSi [32]. YiSi is a family of quality evaluation and estimation metrics for semantic machine translation. In this paper, YiSi-1 is selected for its high average correlation with human assessment, thanks to the use of multilingual bidirectional encoder representations from transformers (BERT).

BLEU, WER, METEOR, ROUGE_L, CIDEr, YiSi were computed using multi-bleu.perl (https://github.com/moses-smt/mosesdecoder), pyter (https://pypi.org/project/pyter/), nlg-eval (METEOR, ROUGE_L, CIDEr using https://github.com/Maluuba/nlg-eval) [34], and YiSi (https://github.com/chikiulo/yisi).

### 4.4. Baselines

1. Original multihead attention by Vaswani et al. [5]: the original transformer-based model is implemented based on multihead attention, which brings more expressive power than single head attention. The model linearly projects the queries, keys, and values with different, learned projection matrices to *d*_*k*_, *d*_*k*_, and *d*_*v*_ dimensions, respectively. Each head yields *d*_*v*_-dimensional output values. All the attention heads are concatenated into the final values.
2. Multihead attention (head size equaling sequence length) by Bhojanapalli et al. [10]: in the original multihead attention, the scaling between the number of heads and head size leads to a low-rank bottleneck. To overcome the problem, Bhojanapalli et al. set the head size to input sequence length and keep it independent of the number of heads. In this way, each head acquires more expressive power. The effectiveness of their approach was verified through experiments on the two tasks of Stanford Question Answering Dataset (SQuAD) and Multigenre Natural Language Inference (MNLI).
3. Talking-head attention by Shazeer et al. [13]: with the increase in the number of heads, the dimensionality of query vectors and key vectors becomes so low that the dot product between the two types of vectors no longer includes useful information. This is what is commonly called a low-rank bottleneck. To address the problem, talking-head attention inserts two linear learned projection matrices across the attention-head dimension of the attention-logits tensor, allowing each head attention to target any subquery vector and subkey vector. The feasibility of this attention mechanism was tested on several seq2seq NLP tasks. But Shazeer et al. did not test the mechanism on any NMT task. Therefore, this paper implements the mechanism on both the evaluation benchmarks and compares it with our model.

### 4.5. Results

For the IWSLT2016 DE-EN translation task, all models almost reached the peak performance at 16 heads. As shown in Table 3, the performance of the original multihead attention clearly declined by 3.31 BLEU/0.41 WER/2.72 METEOR/2.83 ROUGE_L/0.30 CIDEr/3.23 YiSi on the evaluation set and 1.15 WER/2.63 METEOR/2.69 ROUGE_L/0.27 CIDEr/2.88 YiSi on the test set, as the number of heads increased from 16 to 32. The trend signifies the occurrence of the low-rank bottleneck. As for the multihead attention with fixed head size, the performance reached a relatively stable state, when the number of heads was equal to 16. As the number of heads increased, the performance improved slightly. In talking-head attention, the performance varied similarly to multihead attention with fixed head size. When it comes to our interacting-head attention, the performance improved significantly by 2.78 BLEU/0.85 WER/2.90 METEOR/2.65 ROUGE_L/0.29 CIDEr/2.97 YiSi on the evaluation set and 2.43 BLEU/1.38 WER/3.05 METEOR/2.70 ROUGE_L/0.30 CIDEr/3.59 YiSi on the test set, compared with the original multihead attention.

For the WMT17 EN-DE translation task, the original multihead attention had the best performance at 16 heads and performed poorer and poorer with the growing number of heads. As shown in Table 4, multihead attention with fixed head size and talking-head attention achieved a slight improvement by solving the low-rank bottleneck. With our interacting-head attention, the performance improved by 2.31 BLEU/5.94 WER/1.46 METEOR/1.35 ROUGE_L/0.07 CIDEr/0.33 YiSi and 1.62 BLEU/6.04 WER/1.39 METEOR/0.11 CIDEr/0.87 YiSi on the evaluation set and newstest2014, respectively.

For the WMT17 EN-CS translation task, the original multihead attention model once again encountered the low-rank bottleneck at 16 heads. As shown in Table 5, our interacting-head attention achieved better result (3.87 BLEU/3.05 WER/9.22 METEOR/3.81 ROUGE_L/0.36 CIDEr/4.14 YiSi on evaluation set, and 4.62 BLEU/2.41 WER/9.82 METEOR/4.82 ROUGE_L/0.44 CIDEr/5.25 YiSi, 3.78 BLEU/5.09 WER/9.09 METEOR/4.24 ROUGE_L/0.35 CIDEr/3.97 YiSi, 4.42 BLEU/2.87 WER/3.21 METEOR/4.42 ROUGE_L/0.38 CIDEr/4.83 YiSi, and 3.42 BLEU/3.97 WER/2.79 METEOR/3.66 ROUGE_L/0.33 CIDEr/4.00 YiSi on newstest2014/2015/2016/2017, respectively).

### 4.6. Analysis

#### 4.6.1. Horizontal and Longitudinal Analyses

Horizontally, a low-rank bottleneck occurs inevitably, when the number of heads reached a certain level. To some extent, the previous models address this problem at the cost of performance degradation. Machine translation is a generation task between different languages. Compared with the results of previous studies, our model brings significant performance improvement and reveals strong correlations between the subembeddings in different subspaces. Longitudinally, the expressive ability of the model increases with the number of heads, until the latter reaches the bottleneck point **d**/**n**. The superiority of interacting-head attention over the original multihead attention is the result of the function among subembeddings in different subspaces.

#### 4.6.2. Influencing Factor Analysis

As shown in Tables 3 and 4, multihead attention with fixed head size and talking-head attention sacrifice performance for solving the low-rank bottleneck. The final performance is primarily affected by four factors: the dimensions of queries, keys, values, and the number of heads. The leading impactors of the attention matrix are the dimensions of queries and keys. In multihead attention with fixed head size, the attention matrix is realized by the dimensions of queries and keys, both of which are equal to the mean sequence length. The model performance hinges on such factors as the dimension of values, the number of heads, as well as the mean sequence before/after the low-rank bottleneck point. In talking-head attention, the linear transformation has a greater impact on the attention matrix before softmax normalization than after that operation. In our experiments, linear transformations were applied with both functions. The poor performance may be attributable to the use of masked multihead attention in the decoder.

Interacting-head attention is more effective than the original multihead attention, revealing a strong relationship between the head size of different subspaces. Specifically, when the number of heads is small, there is a strong relationship between different subembeddings in different subspaces. With the growth of the number of heads, the said relationship is gradually weakened. In particular, interacting-head attention degenerates into multihead attention, after the number of heads surpasses d/n.

#### 4.6.3. Training Speed

As shown in Figures 4–6 and Tables 6–8, the training time of our model extended significantly when there were 16 heads. The value of 8 was selected to strike a balance between the training time and the decoding performance. In particular, for the IWSLT16 DE-EN dataset, the training time per epoch of our model increased by only 13 minutes, while the performance was improved by 2 BLEU. The slowdown of training is caused by the calculation of the attention relationship among different subspaces.

#### 4.6.4. Trainable Variables

Compared with the original multihead attention, the interacting-head attention model does not bring more training parameters but only adds the inner product calculation of tensors in different subspaces. The tensor calculation of different tokens in different subspaces slows down the training process. The slowdown is no big deal, given the huge translation improvement of our model. Besides, this problem can be solved by setting the maximum number of heads as a fixed scalar.

#### 4.6.5. Maximum Number of Heads

To verify the suitability of the number of heads, our model was subjected to an ablation test, with the number of heads changing from 32 to 64. As shown in Table 9, a low-rank bottleneck occurred, once the number of heads exceeded a threshold, although the performance of our model was better than that of the original multihead attention. According to the performance variation, the threshold should be **d**/**n** as the maximum number of heads. The test was only carried out on the IWSLT16 DE-EN dataset because the training time of our model grows exponentially after the number of heads surpasses the threshold.

### 4.7. Discussion

In original multihead attention, the translation performance is positively correlated with the number of heads when the heads are between 2 and 16 and negatively correlated with the number of heads when the heads surpass 16. Within a certain range, many heads enhance the expressive power. Once the number exceeds a threshold, a low-rank bottleneck will take place, due to the ultrasmall dimensionality in the subspace. In original multihead attention, when there are many heads, the dimensions of each subquery, subkey, and subvalue meet the condition: *d*_*q*_=*d*_*k*_=*d*_*v*_=*d*_model_/*h*. In this case, *d*_*q*_ and *d*_*k*_ are small, and the sequence length is usually greater than *d*_model_/*h*.

In multihead attention with fixed head size, the low-rank bottleneck can be avoided by setting *d*_*q*_=*d*_*k*_=*n* in the subspace, when there are many heads.

In talking-head attention, the independence of the subattention matrices is improved through linear transformation between the subhead attention matrices, which is actually performed between the *i* − *thd*_*q*_ and the *j* − *thd*_*k*_. However, the attention matrices in the sequences are actually sparse. The sparsity can be inferred through the syntactic dependency tree and Bayesian network, and even be observed through visualization tools like Bertviz [35] (https://github.com/jessevig/bertviz). The irregular sparsity makes it difficult to learn the optimal weight coefficients from the overall perspective of the attention matrix.

In our model, two thorny problems are resolved. Firstly, the original multihead attention only calculates the hidden features of different tokens in the same space and concatenates all subfeatures into the final output. However, our experimental results show certain connections of different tokens in different subspaces. Secondly, our model adopts the solution of multihead attention with fixed head size and proposes a method for optimizing the maximum number of heads, thereby preventing the low-rank bottleneck induced by the low dimensionality of the subspaces. The disadvantage of our model is the requirement of many tensor calculations, which prolongs the training time. Future research will try to reduce the tensor calculations by capturing the key attention and ignoring the minor attention between the tokens.

## 5. Conclusion

Currently, the transformer-based models employ the multihead attention mechanism for NMT, which computes the attention scores between the tokens themselves and among the tokens in the same subspaces. However, language is complex, which contains multidimensional information such as lexical, syntactic, and semantic information, and there are relationships between different dimensions of information. Therefore, this paper proposes the interacting-head attention model, which boasts two advantages. On the one hand, our model confirms the attention relationship between different tokens in different subspaces and uses this relationship to improve translation performance. On the other hand, the model provides a new method for optimizing the maximum number of heads, which helps to prevent the low-rank bottleneck. Besides, a threshold was defined for the number of heads, aiming to avoid the exponential growth of training time. Under this premise, using our model can greatly improve the translation performance. In conclusion, experimental research in this paper argues that the interacting-head attention mechanism is significantly effective for NMT. Simultaneously, the experimental results show that there is a strong interaction in the different dimensions of information of all the tokens within a sequence.

However, this model has 2 disadvantages. On the one hand, the attention scores between sequence tokens are different, and some even tend to be 0. Therefore, the attention relationship between tokens should not be a fully connected network, but a sparse network which also can reduce the time complexity of computing the attention matrix. On the other hand, considering the attention relationship between different tokens in different subspaces, it is necessary to perform lots of tensor inner product calculations, especially with more heads. As a result, the training and decoding times are extended to a certain extent. These defects of the proposed model will be addressed in future work.

## Figures and Tables

**Figure 1:** Associations between the head size of different subspaces.

**Figure 2:** Comparison between multihead attention (a) and our mechanism (b) with 4 heads.

**Figure 3:** Histogram and line graph of sequence length distribution of IWSLT16 DE-EN, WMT17 EN-DE, and WMT17 EN-CS.

**Figure 4:** Training time of each epoch of four models on the IWSLT16 DE-EN dataset.

**Figure 5:** Training time of each epoch of four models on the WMT17 EN-DE dataset.

**Figure 6:** Training time of each epoch of four models on WMT17 EN-CS dataset.

**Algorithm 1:** Interacting-head Attention.

**Table 1:** Number of sequence pairs and sequence length in IWSLT16 DE-EN, WMT17 EN-DE, and WMT17 EN-CS.

Dataset	Train	Eval	Test	Vocab	Total length of the train set	Mean length of the train set
IWSLT16 DE-EN	181,149	12,098	11,825	39,645	3,766,897/3,826,038	20/21
WMT17 EN-DE	5,852,457	3000	3003/2169/2999/3004	84,441	148,665,327/149,176,205	25/25
WMT17 EN-CS	1,010,918	3000	3003/2656/2999/3005	25,560/39,670	27,825,644/26,152,299	27/25

*Note.* Train, Eval, and Test represent the number of sequence pairs of different data subsets, respectively; length refers to the number of tokens in a sentence; total length of the train set is the total number of tokens in the training set; mean length of the train set is the ratio of the total length to the total sequence pairs in the training set.

**Table 2:** Possible number of heads in our model.

Dataset	Model	Number of heads
IWSLT16 DE-EN	512	25 [2, 4, 8, 16]
WMT17 EN-DE	512	20 [2, 4, 8, 16]
WMT17 EN-CS	512	20 [2, 4, 8, 16]

**Table 3:** Overall evaluation scores using four attention-based models on the IWSLT16 DE-EN evaluation set and test set.

Model	IWSLT16 subset	Number of heads/Head size					
		2/256	4/128	8/64	16/32	32/16	64/8
*(a)*							
Multihead attention	dev	22.73	25.71	26.44	**27.23**	23.92	19.50
	Test	21.15	24.00	24.38	**25.18**	22.05	17.94
Multihead attention (head size = *n*, dmodel = 512)	dev	20.93	23.08	24.79	26.00	**26.94**	26.38
	Test	19.35	21.38	22.81	24.61	**24.86**	24.59
Talking-head attention	dev	20.66	21.39	22.47	24.02	**24.21**	23.65
	Test	19.13	19.82	20.87	22.24	**22.30**	21.72
Interacting-head attention	dev	29.59	29.94	29.54	**30.01(+2.78)**	—	—
	Test	27.61	28.01	27.44	**27.61(+2.43)**	—	—

*(b)*							
Multihead attention	dev	5.82	4.85	3.56	**3.10**	3.51	8.73
	Test	9.03	7.92	7.71	**5.87**	7.02	14.39
Multihead attention (head size = *n*, dmodel = 512)	dev	6.90	6.00	5.29	4.59	4.55	**3.97**
	Test	11.47	10.10	8.98	8.16	8.11	**7.96**
Talking-head attention	dev	9.03	7.31	6.58	4.81	4.51	**4.33**
	Test	14.46	11.90	9.83	9.10	**8.69**	8.90
Interacting-head attention	dev	2.41	2.44	2.31	**2.25(0.85)**	—	—
	Test	6.60	5.34	4.77	**4.49(1.38)**	—	—

*(c)*							
Multihead attention	dev	25.42	26.72	28.58	**29.14**	26.42	22.63
	Test	24.77	25.96	27.67	**28.20**	25.57	22.02
Multihead attention (head size = *n*, dmodel = 512)	dev	23.47	25.69	25.76	26.51	27.05	**27.12**
	Test	22.84	24.95	24.95	25.88	25.28	**26.36**
Talking-head attention	dev	22.48	24.28	23.80	24.46	25.28	**26.76**
	Test	21.85	23.46	23.18	23.94	24.49	**25.85**
Interacting-head attention	dev	31.73	31.94	31.65	**32.04(+2.90)**	—	—
	Test	30.87	31.11	30.76	**31.25(+3.05)**	—	—

*(d)*							
Multihead attention	dev	53.72	55.68	57.85	**58.76**	55.93	50.52
	Test	52.23	54.30	56.23	**57.26**	54.57	49.24
Multihead attention (head size = *n*, dmodel = 512)	dev	51.46	54.02	55.83	55.52	56.53	**56.99**
	Test	50.21	52.70	55.44	54.31	54.18	**55.60**
Talking-head attention	dev	49.26	51.64	52.38	53.72	54.92	**55.78**
	Test	48.23	50.19	51.19	52.30	53.33	**54.45**
Interacting-head attention	dev	61.02	61.29	61.14	**61.41(+2.65)**	—	—
	Test	59.25	59.80	59.62	**59.96(+2.70)**	—	—

*(e)*							
Multihead attention	dev	1.94	2.39	2.61	**2.69**	2.39	1.89
	Test	1.80	2.20	2.39	**2.49**	2.22	1.75
Multihead attention (head size = *n*, dmodel = 512)	dev	1.99	2.20	2.24	2.27	2.33	**2.38**
	Test	1.84	2.05	2.08	2.10	2.16	**2.21**
Talking-head attention	dev	1.70	1.87	1.84	2.09	2.20	**2.32**
	Test	1.57	1.72	1.67	1.91	2.01	**2.05**
Interacting-head attention	dev	2.93	2.96	2.93	**2.98(+0.29)**	—	—
	Test	2.69	2.75	2.71	**2.79(+0.30)**	—	—

*(f)*							
Multihead attention	dev	54.33	55.98	57.91	**58.48**	55.25	49.83
	Test	53.34	54.18	55.88	**56.45**	53.57	48.44
Multihead attention (head size = *n*, dmodel = 512)	dev	52.05	54.25	55.85	57.15	**57.33**	56.45
	Test	50.63	52.57	54.18	55.51	**56.79**	55.94
Talking-head attention	dev	50.19	51.32	52.32	53.02	55.55	**57.06**
	Test	48.97	49.63	50.63	51.69	53.72	**55.83**
Interacting-head attention	dev	60.92	61.22	60.91	**61.45(+2.97)**	—	—
	Test	58.68	59.15	58.67	**60.04(+3.59)**	—	—

*Note.* The units of the performances are (a) BLEU, (b) WER, (c) METEOR, (d) ROUGE_L, (e) CIDEr, and (f) YiSi.

**Table 4:** Overall evaluation scores using four attention-based models on the WMT17 EN-DE evaluation set and test set.

Model	WMT17 subset	Number of heads/head size					
		2/256	4/128	8/64	16/32	32/16	64/8
*(a)*							

Multihead attention	dev	8.38	12.56	12.48	**15.15**	12.20	12.45
	newstest2014	8.77	11.31	12.85	**15.73**	11.61	12.28
	newstest2015	9.36	12.27	13.80	**16.79**	11.90	13.23
	newstest2016	11.40	14.83	16.79	**20.97**	15.17	16.16
	newstest2017	8.83	11.83	13.15	**16.41**	11.63	12.99

Multihead attention (head size = *n*)	dev	11.66	12.51	13.70	14.57	14.61	**15.29**
	newstest2014	11.64	13.26	14.93	**15.42**	14.96	15.00
	newstest2015	12.04	14.07	15.78	16.57	16.67	**17.57**
	newstest2016	14.71	17.57	19.77	**20.33**	19.80	20.08
	newstest2017	11.72	13.54	14.92	16.03	16.07	**16.33**

Talking-head attention	dev	10.90	13.89	15.31	15.37	15.23	**15.50**
	newstest2014	11.21	12.64	14.33	15.28	15.29	**15.39**
	newstest2015	11.85	12.81	14.61	**15.95**	15.55	15.36
	newstest2016	14.22	16.33	18.84	19.53	19.34	**20.43**
	newstest2017	11.15	12.81	14.35	**15.49**	14.44	15.36

Interacting-head attention	dev	13.07	14.84	14.53	**17.46(+2.31)**	—	—
	newstest2014	10.91	14.72	15.75	**17.35(+1.62)**	—	—
	newstest2015	11.99	15.43	16.90	**18.40(+1.21)**	—	—
	newstest2016	14.95	19.61	21.12	**22.36(+1.39)**	—	—
	newstest2017	11.09	15.00	17.30	**17.67(+1.26)**	—	—

*(b)*							

Multihead attention	dev	39.23	37.80	28.23	**15.57**	32.93	22.47
	newstest2014	46.85	45.59	32.10	**19.68**	39.59	28.80
	newstest2015	45.22	44.31	32.64	**22.68**	42.78	28.58
	newstest2016	40.14	39.35	28.51	**15.91**	32.04	23.97
	newstest2017	43.85	42.74	32.12	**19.07**	38.38	26.50

Multihead attention (head size = *n*)	dev	39.37	36.73	25.11	22.97	16.67	**13.42**
	newstest2014	46.40	35.77	32.56	28.65	**18.56**	18.77
	newstest2015	46.93	38.45	33.16	28.03	23.13	**20.07**
	newstest2016	42.91	30.24	27.66	22.77	17.15	**13.26**
	newstest2017	44.65	34.60	29.82	26.78	19.75	**16.52**

Talking-head attention	dev	48.17	40.63	39.03	24.80	20.13	**16.25**
	newstest2014	48.19	48.02	52.98	33.93	27.58	**20.32**
	newstest2015	61.09	53.80	52.33	33.43	31.13	**22.05**
	newstest2016	47.02	47.28	47.42	31.08	23.16	**14.82**
	newstest2017	51.13	47.34	50.63	34.52	28.01	**20.05**

Interacting-head attention	dev	58.10	35.20	20.83	**9.63(5.94)**	—	—
	newstest2014	68.39	47.29	29.01	**13.64(6.04)**	—	—
	newstest2015	79.39	48.55	29.64	**16.05(6.63)**	—	—
	newstest2016	67.12	44.21	25.94	**11.27(4.64)**	—	—
	newstest2017	81.56	49.07	30.89	**15.23(3.84)**	—	—

*(c)*							

Multihead attention	dev	19.36	19.54	20.31	**23.16**	20.56	20.53
	newstest2014	19.39	19.64	20.83	**23.71**	20.72	20.97
	newstest2015	19.36	19.60	21.15	**24.11**	20.70	21.06
	newstest2016	20.43	21.27	22.73	**26.29**	22.44	22.63
	newstest2017	19.52	19.85	21.05	**23.96**	20.70	21.11

Multihead attention (head size = *n*)	dev	19.47	20.96	21.04	23.01	23.32	**23.79**
	newstest2014	19.69	21.45	22.30	23.52	23.91	**24.45**
	newstest2015	19.64	21.54	22.61	23.70	24.02	**24.46**
	newstest2016	20.95	23.26	24.47	25.65	25.44	**26.99**
	newstest2017	19.68	21.50	22.25	23.73	24.05	**24.49**

Talking-head attention	dev	17.71	19.55	21.38	23.22	**23.51**	23.19
	newstest2014	17.73	19.59	21.87	23.65	23.73	**23.75**
	newstest2015	17.33	19.39	22.03	23.81	24.14	**24.26**
	newstest2016	18.60	20.52	23.19	25.40	**26.02**	25.88
	newstest2017	17.74	19.39	21.90	23.71	23.66	**24.15**

Interacting-head attention	dev	22.43	22.61	23.87	**24.62(+1.46)**	—	—
	newstest2014	22.67	22.66	24.35	**25.10(+1.39)**	—	—
	newstest2015	22.81	23.09	24.52	**25.53(+1.42)**	—	—
	newstest2016	24.69	25.00	26.68	**27.27(+0.98)**	—	—
	newstest2017	22.12	22.76	24.38	**25.66(+1.70)**	—	—

*(d)*							

Multihead attention	dev	40.08	40.19	41.54	**45.77**	42.47	42.79
	newstest2014	36.65	37.81	40.22	**49.04**	40.40	41.18
	newstest2015	37.33	39.63	42.56	**46.84**	41.69	42.71
	newstest2016	39.88	41.98	44.40	**44.88**	44.52	45.13
	newstest2017	36.94	39.01	41.43	**46.09**	41.02	42.02

Multihead attention (head size = *n*)	dev	41.39	43.67	44.89	45.79	45.83	**46.01**
	newstest2014	39.75	42.35	43.62	44.69	45.07	**47.25**
	newstest2015	40.76	43.37	45.54	46.18	46.22	**48.15**
	newstest2016	43.18	46.51	48.21	49.34	48.96	**50.08**
	newstest2017	40.41	43.05	44.87	45.52	45.55	**46.08**

Talking-head attention	dev	38.42	40.20	42.03	43.99	44.67	**45.33**
	newstest2014	35.67	39.23	42.51	42.74	45.86	**46.09**
	newstest2015	37.94	38.61	41.00	44.15	44.92	**46.67**
	newstest2016	38.83	41.21	42.88	46.28	**48.05**	46.99
	newstest2017	37.29	39.58	40.93	43.30	45.23	**45.65**

Interacting-head attention	dev	45.47	46.03	46.54	**47.12(+1.35)**	—	—
	newstest2014	43.95	43.77	45.15	**48.20**	—	—
	newstest2015	45.33	45.83	46.61	**47.31(+0.51)**	—	—
	newstest2016	47.97	48.83	49.94	**50.47(+5.59)**	—	—
	newstest2017	43.61	44.58	45.91	**45.99**	—	—

*(e)*							

Multihead attention	dev	1.26	1.30	1.37	**1.64**	1.37	1.38
	newstest2014	1.13	1.19	1.26	**1.52**	1.26	1.26
	newstest2015	1.24	1.31	1.42	**1.63**	1.36	1.36
	newstest2016	1.39	1.50	1.62	**1.93**	1.61	1.60
	newstest2017	1.17	1.22	1.35	**1.61**	1.29	1.33

Multihead attention (head size = *n*)	dev	1.23	1.38	1.45	1.63	1.63	**1.66**
	newstest2014	1.13	1.30	1.39	1.54	1.55	**1.58**
	newstest2015	1.19	1.37	1.45	1.67	**1.68**	1.65
	newstest2016	1.38	1.65	1.80	1.94	1.85	**1.99**
	newstest2017	1.16	1.35	1.43	1.60	**1.71**	1.70

Talking-head attention	dev	1.06	1.20	1.38	1.42	1.49	**1.58**
	newstest2014	0.96	1.11	1.35	1.38	1.46	**1.51**
	newstest2015	1.04	1.20	1.37	1.39	1.36	**1.39**
	newstest2016	1.16	1.40	1.67	1.45	1.48	**1.62**
	newstest2017	0.98	1.15	1.43	1.39	**1.48**	1.47

Interacting-head attention	dev	1.63	1.64	1.67	**1.71(+0.07)**	—	—
	newstest2014	1.43	1.51	1.57	**1.63(+0.11)**	—	—
	newstest2015	1.63	1.61	1.74	**1.81(+0.18)**	—	—
	newstest2016	1.89	1.88	2.02	**2.17(+0.24)**	—	—
	newstest2017	1.52	1.50	1.65	**1.74(+0.13)**	—	—

*(f)*							

Multihead attention	dev	43.74	44.71	45.35	**48.82**	46.28	45.37
	newstest2014	41.50	42.57	43.80	**47.84**	44.44	43.77
	newstest2015	43.17	44.10	45.99	**49.68**	45.81	45.49
	newstest2016	44.90	45.96	47.37	**52.29**	47.86	47.13
	newstest2017	42.11	43.36	44.99	**48.71**	44.91	44.71

Multihead attention (head size = *n*)	dev	44.58	46.00	47.06	48.51	48.99	**49.01**
	newstest2014	43.09	44.63	45.63	47.40	48.04	47.99
	newstest2015	44.37	46.09	47.54	48.83	49.15	**49.56**
	newstest2016	46.24	48.30	49.65	51.20	51.30	51.06
	newstest2017	43.82	45.47	46.38	48.34	48.55	**48.77**

Talking-head attention	dev	38.11	39.63	40.73	44.07	46.14	**48.60**
	newstest2014	35.46	38.32	39.02	42.77	44.52	**47.33**
	newstest2015	**37.48**	38.71	40.35	44.35	46.84	49.52
	newstest2016	37.09	40.25	41.43	45.96	48.36	**50.70**
	newstest2017	**36.20**	38.93	39.47	43.75	45.85	48.05

Interacting-head attention	dev	48.03	48.23	48.78	**49.15(+0.33)**	—	—
	newstest2014	46.72	46.63	47.78	**48.71(+0.87)**	—	—
	newstest2015	48.11	48.52	49.09	**50.20(+0.52)**	—	—
	newstest2016	50.88	50.77	51.47	**52.71(+0.42)**	—	—
	newstest2017	47.73	48.48	49.83	**50.01(+1.30)**	—	—

*Note.* The units of the performances are (a) BLEU, (b) WER, (c) METEOR, (d) ROUGE_L, (e) CIDEr, and (f) YiSi.

**Table 5:** Overall evaluation scores using four attention-based models on the WMT17 EN-CS evaluation set and test set.

Model	WMT17 subset	Number of heads/head size					
		2/256	4/128	8/64	16/32	32/16	64/8
*(a)*							

Multihead attention	dev	11.69	13.96	13.76	**14.14**	12.10	11.98
	newstest2014	12.90	15.65	14.82	**15.52**	13.26	12.71
	newstest2015	11.03	12.48	11.66	**12.62**	10.04	10.08
	newstest2016	11.98	13.85	13.09	**14.32**	11.16	10.85
	newstest2017	10.26	12.45	11.71	**12.36**	9.96	10.14

Multihead attention (head size = *n*)	dev	10.14	11.87	12.99	13.35	14.36	14.46
	newstest2014	11.32	13.34	14.04	14.49	15.79	15.28
	newstest2015	9.11	10.18	11.55	11.67	12.69	12.05
	newstest2016	10.23	11.86	12.51	12.62	13.73	13.83
	newstest2017	8.99	10.43	11.30	11.23	12.54	12.47

Talking-head attention	dev	9.80	10.06	11.77	12.06	12.75	12.68
	newstest2014	10.90	10.65	11.65	12.33	12.94	12.34
	newstest2015	8.17	8.54	10.06	11.70	11.51	11.57
	newstest2016	9.11	9.38	10.50	11.25	11.78	11.73
	newstest2017	8.50	8.63	9.92	11.05	11.52	11.83

Interacting-head attention (our model)	dev	17.01	17.76	17.93	**18.01(+3.87)**	—	—
	newstest2014	18.71	19.48	20.01	**20.14(+4.62)**	—	—
	newstest2015	15.52	**16.49**	16.38	16.40(+3.78)	—	—
	newstest2016	17.20	18.37	18.29	**18.74(+4.42)**	—	—
	newstest2017	14.66	15.66	15.79	**15.78(+3.42)**	—	—

*(b)*							

Multihead attention	dev	15.13	12.33	15.27	**10.30**	29.60	16.80
	newstest2014	13.95	11.66	14.15	**8.62**	25.57	13.85
	newstest2015	23.68	17.96	23.34	**17.17**	39.53	24.06
	newstest2016	18.44	14.90	19.31	**12.70**	35.28	21.31
	newstest2017	20.70	18.20	21.06	**16.21**	36.44	21.63

Multihead attention (head size = *n*)	dev	17.30	15.53	13.43	12.43	**10.83**	14.37
	newstest2014	15.02	14.35	12.12	11.12	9.19	**8.56**
	newstest2015	27.60	23.87	20.22	18.71	**16.79**	16.91
	newstest2016	21.34	20.34	18.24	16.24	**13.80**	14.37
	newstest2017	24.23	21.56	20.07	19.27	**15.91**	18.66

Talking-head attention	dev	28.37	43.43	**27.00**	34.33	27.57	27.51
	newstest2014	21.25	33.70	28.94	34.97	25.86	**26.22**
	newstest2015	38.03	55.35	**37.95**	47.21	42.48	46.87
	newstest2016	30.31	45.82	**34.44**	44.11	36.35	36.83
	newstest2017	31.01	47.75	35.77	41.63	35.86	**35.76**

Interacting-head attention (our model)	dev	7.63	7.27	8.03	**7.25(3.05)**	—	—
	newstest2014	6.99	6.43	7.16	**6.21(2.41)**	—	—
	newstest2015	12.99	12.09	11.94	**12.08(5.09)**	—	—
	newstest2016	10.14	**9.80**	9.70	9.83(2.87)	—	—
	newstest2017	12.48	12.95	**11.71**	12.24(3.97)	—	—

*(c)*							

Multihead attention	dev	17.37	19.52	19.16	**19.55**	18.85	17.92
	newstest2014	18.41	**20.82**	20.42	20.80	19.92	18.93
	newstest2015	16.69	**18.90**	18.51	18.77	18.17	17.32
	newstest2016	17.21	**19.59**	19.05	19.36	18.44	17.45
	newstest2017	15.65	**17.96**	17.51	17.85	17.13	16.26

Multihead attention (head size = *n*)	dev	16.09	17.62	18.65	18.91	**19.68**	18.10
	newstest2014	17.04	18.82	19.69	20.09	**20.88**	20.06
	newstest2015	15.30	16.68	18.08	18.16	**19.05**	18.37
	newstest2016	15.85	17.42	18.41	18.62	**19.39**	18.92
	newstest2017	14.70	16.00	16.99	17.10	**19.99**	17.42

Talking-head attention	dev	15.93	15.82	16.05	**16.85**	16.48	16.72
	newstest2014	16.86	16.58	16.33	**17.04**	16.76	16.76
	newstest2015	15.00	14.74	14.97	15.75	15.68	**16.12**
	newstest2016	15.59	15.08	15.07	**15.87**	15.50	15.85
	newstest2017	14.33	14.01	14.11	15.15	14.87	**15.62**

Interacting-head attention	dev	21.76	22.43	25.90	**28.77(+9.22)**	—	—
	newstest2014	23.30	24.28	28.07	**30.62(+9.82)**	—	—
	newstest2015	21.08	21.98	25.28	**27.86(+9.09)**	—	—
	newstest2016	21.99	**22.95**	21.98	22.57(+3.21)	—	—
	newstest2017	19.81	20.55	19.72	**20.64(+2.79)**	—	—

*(d)*							

Multihead attention	dev	39.80	43.15	42.51	**43.27**	41.93	40.36
	newstest2014	41.25	44.98	44.22	**45.14**	43.31	42.08
	newstest2015	39.04	42.13	41.42	**42.20**	40.74	39.46
	newstest2016	39.00	42.82	41.81	**42.82**	40.41	39.08
	newstest2017	37.29	40.34	39.80	**40.46**	38.83	37.75

Multihead attention (head size = *n*)	dev	37.50	40.03	41.71	42.17	**43.36**	43.13
	newstest2014	38.90	41.91	43.11	43.66	**44.95**	44.47
	newstest2015	36.23	38.51	40.99	40.83	**42.40**	41.67
	newstest2016	36.87	39.16	40.81	40.99	**42.41**	42.19
	newstest2017	35.11	37.52	38.95	38.94	**40.59**	40.38

Talking-head attention	dev	36.01	37.56	38.58	40.74	**41.37**	40.95
	newstest2014	37.76	39.21	38.36	40.42	**41.46**	41.27
	newstest2015	34.23	35.22	36.80	39.02	40.06	**40.81**
	newstest2016	35.10	36.06	36.42	38.53	39.47	**39.9**5
	newstest2017	33.50	34.71	35.46	37.76	**38.62**	38.41

Interacting-head attention (our model)	dev	46.07	45.90	46.87	**47.08(+3.81)**	—	—
	newstest2014	48.17	48.07	49.13	**49.96(+4.82)**	—	—
	newstest2015	45.22	45.28	46.01	**46.44(+4.24)**	—	—
	newstest2016	45.87	45.94	46.87	**47.24(+4.42)**	—	—
	newstest2017	42.83	42.93	43.65	**44.12(+3.66)**	—	—

*(e)*							

Multihead attention	dev	**1.42**	1.38	1.37	1.40	1.32	1.20
	newstest2014	1.24	1.53	1.47	**1.56**	1.44	1.30
	newstest2015	1.09	1.30	1.27	**1.32**	1.24	1.11
	newstest2016	1.10	1.37	1.30	**1.37**	1.23	1.11
	newstest2017	1.02	1.22	1.20	1.25	**1.44**	1.06

Multihead attention (head size = *n*)	dev	1.01	1.18	1.29	1.32	1.42	**1.44**
	newstest2014	1.07	1.29	1.39	1.44	1.53	**1.53**
	newstest2015	0.91	1.06	1.22	1.22	**1.32**	1.31
	newstest2016	0.96	1.12	1.23	1.27	1.35	**1.37**
	newstest2017	0.88	1.03	1.14	**1.35**	1.25	1.28

Talking-head attention	dev	0.90	0.74	0.92	0.80	0.79	
	newstest2014	0.99	0.81	0.92	0.79	0.78	0.34
	newstest2015	0.79	0.63	0.90	0.70	0.70	0.32
	newstest2016	0.83	0.67	0.78	0.69	0.69	0.30
	newstest2017	0.78	0.61	0.77	0.68	0.67	0.33

Interacting-head attention	dev	1.63	**1.74(+0.36)**	1.64			
	newstest2014	1.79	**1.97(+0.44)**	1.80			
	newstest2015	1.55	**1.65(+0.35)**	1.56			
	newstest2016	1.62	**1.75(+0.38)**	1.64			
	newstest2017	1.43	**1.55(+0.33)**	1.47			

*(f)*							

Multihead attention	dev	28.64	**32.37**	31.74	32.12	31.41	29.07
	newstest2014	30.37	**34.58**	33.72	34.47	33.02	31.14
	newstest2015	27.67	**31.15**	30.47	30.93	30.13	28.24
	newstest2016	28.10	**32.11**	31.22	31.89	30.07	28.22
	newstest2017	26.20	**29.89**	29.24	29.54	28.53	26.80

Multihead attention (head size = *n*)	dev	26.65	28.94	30.62	31.06	32.26	**32.57**
	newstest2014	28.00	31.21	32.42	32.99	34.23	**34.23**
	newstest2015	25.02	27.25	29.69	29.68	**31.07**	31.05
	newstest2016	25.80	28.29	30.02	30.27	31.50	**31.75**
	newstest2017	24.27	26.59	28.11	28.11	29.76	**30.05**

Talking-head attention	dev	25.19	27.48	29.82	30.23	**31.50**	31.47
	newstest2014	27.12	29.28	29.94	30.20	31.75	**31.82**
	newstest2015	23.60	25.37	27.98	28.57	30.17	**30.55**
	newstest2016	24.51	26.37	28.09	28.39	**29.68**	29.64
	newstest2017	22.79	24.89	26.90	27.37	28.81	**28.88**

Interacting-head attention	dev	35.34	35.09	36.50	**36.51(+4.14)**	—	—
	newstest2014	37.77	37.59	38.75	**39.83(+5.25)**	—	—
	newstest2015	34.32	34.25	35.17	**35.48(+3.97)**	—	—
	newstest2016	35.28	35.39	35.68	**36.94(4.83)**	—	—
	newstest2017	32.40	32.58	**34.81**	33.89(+4.00)	—	—

*Note.* The units of the performances are (a) BLEU, (b) WER, (c) METEOR, (d) ROUGE_L, (e) CIDEr, and (f) YiSi.

**Table 6:** Training time on IWSLT16 DE-EN training dataset.

Model	Number of heads					
	2	4	8	16	32	64
Multihead attention	10 m 10 s	10 m 30 s	10 m 55 s	11 m 30 s	12 m 45 s	15 m 30 s
Multihead attention (head size = *n*)	9 m 20 s	9 m 40 s	10 m 10 s	11 m 05 s	12 m 55 s	16 m 55 s
Talking-head attention	10 m 30 s	10 m 40 s	11 m	11 m 40 s	15 m 50 s	
Interacting-head attention	10 m 30 s	11 m 30 s	14 m 30 s	24 m 30 s	—	—

*Note.* The units of m and s stand for minute and second, respectively.

**Table 7:** Training time on WMT17 EN-DE training dataset.

Model	Number of heads/head size					
	2/256	4/128	8/64	16/32	32/16	64/8
Multihead attention	9 h 55 m	11 h	11 h 30 m	12 h	12 h 30 m	14 h
Multihead attention (head size = *n*)	11 h 30 m	11 h 40 m	11 h 50 m	12 h 50 m	13 h 10 m	17 h 30 m
Talking-head attention	11 h 5 m	11 h 40 m	11 h 50 m	12 h 20 m	13 h 50 m	15 h
Interacting-head attention	10 h 40 m	11 h 30 m	12 h 50 m	20 h	—	—

*Note.* The units of h, m, and s stand for hour, minute, and second, respectively.

**Table 8:** Training time on the WMT17 EN-CS training dataset.

Model	Number of heads/head size					
	2/256	4/128	8/64	16/32	32/16	64/8
Multihead attention	1 h	1 h 5 m	1 h 8 m	1 h 10 m	1 h 15 m	1 h 30 m
Multihead attention (head size = *n*)	50 m	53 m	57 m	1 h 3 m	1 h 15 m	1 h 50 m
Talking-head attention	58 m	59 m	1 h	1 h 5 m	1 h 10 m	1 h 30 m
Interacting-head attention	53 m	58 m	1 h 13 m	1 h 50 m	—	—

*Note.* The units of h, m, and s stand for hour, minute, and second, respectively.

**Table 9:** Overall evaluation scores of interacting-head attention on IWSLT16 DE-EN evaluation set and test set.

Model	Dataset	Subset	Number of heads/head size	
			32/16	64/8
Interacting-head attention	**IWSLT16**	dev	24.38	19.98
		Test	22.85	18.54

*Note.* The unit of the performance is BLEU.

## Data Availability

The data that support the findings of this study are publicly available from https://wit3.fbk.eu and https://www.statmt.org/wmt17/translation-task.html. If the IWSLT16 DE-EN corpus is used in your work, reference [18] should be cited. If the WMT17 EN-DE and EN-CS corpora are used in your work, references [19, 20] should be cited.
